RETRACTED

# Rapid screening system to identify unspecific peroxygenase activity*

**DOI:** 10.1177/13860291241306566

**Published:** 2025-04-27

**Authors:** Marina Schramm, Carlos Renato Carrillo Avilés, Johannes Kalmbach, Kai-Uwe Schmidtke, Jan Kiebist, Harald Kellner, Martin Hofrichter, Katrin Scheibner

**Affiliations:** 1 Institute of Biotechnology, Brandenburg University of Technology Cottbus-Senftenberg, Senftenberg, Germany; 2 Fraunhofer Institute for Cell Therapy and Immunology, Branch Bioanalytics and Bioprocesses, Potsdam-Golm, Germany; 3 Department of Bio- and Environmental Sciences, TU Dresden-International Institute Zittau, Zittau, Germany

**Keywords:** screening assay, ABTS, unspecific peroxygenase, drug metabolism, enzyme expression, omega-3-lipids metabolism

## Abstract

Unspecific peroxygenases (UPO, EC 1.11.2.1) are a valuable tool for the biocatalytic synthesis of specialty chemicals such as pharmaceutical metabolites. However, the search for new UPOs that are recombinantly expressible can be tedious and dependent on expensive equipment, especially when a large number of clones has to be examined. In this study, we present a simple agar plate-based method for the screening of active, secreted UPOs heterologously expressed in *Saccharomyces cerevisiae*. This allows a real high-throughput of several thousand clones at once. The approach was successfully tested with a small gene library comprising putative UPO genes and resulted in the identification of two clones producing short UPOs from the filamentous fungi *Dendrothele bispora* (*Dbi*UPO) and *Aspergillus niger* (*Ani*UPO). Both UPOs were partly purified and characterized with respect to their catalytic properties. With differing efficiencies and product specificities, they catalyzed the formation of human drug metabolites, e.g., lipid mediators from polyunsaturated fatty acids and the active metabolite of the prodrug clopidogrel, respectively.

## Introduction

There is a great need for new or chemically modified low-molecular platelet aggregation inhibitors, but also for drugs with fewer unwanted interaction and adverse effects on endothelial function or the haematopoietic system in order to reduce complications such as venous thrombosis or arterial occlusion.^1–4^ We were interested in investigating a biotechnological approach to identify enzymes that could modify common (pro-)drugs such as clopidogrel to produce human-like metabolites that could be used in diagnostics or pharmacy.

Unspecific peroxygenases (UPO, EC 1.11.2.1) are secreted enzymes that are found in numerous fungi and have a unique potential for applications in organic synthesis. They are able to selectively incorporate peroxide-borne oxygen into activated and non-activated hydrocarbons, leading to hydroxylations and epoxidations, which are difficult to realize by chemical methods.^5–8^ However, their reaction portfolio does not only include P450-like monooxygenase but also peroxidase activities.^9^ Particularly valuable is the use of UPOs in the synthesis of pharmaceutical metabolites:^10^ thus, they have successfully been used in the preparation of human drug metabolites from different substance classes, for example, from polyunsaturated fatty acids (PUFAs),^11^ propranolol,^12,13^ and from prodrugs such as clopidogrel.^14^ In addition, they are useful to synthesize active pharmaceutical ingredients,^15^ which altogether shows their suitability for diagnostics and drug development.

RETRACTED

Extensive sequencing of fungal genomes over the last years and metagenomic approaches revealed the existence of thousands of putative UPO genes in most phylogenetic groups of fungi.^9^ Since each UPO has its own catalytic portfolio, there is an immense reservoir for specific biocatalysts to be used in organic synthesis. However, the identification of new UPOs that can be produced in adequate quantities remains a challenge, whether in the original organism or in a heterologous host. An overview of successful approaches for the production of UPOs was provided in the review article by Kinner et al. from 2021;^16^ the corresponding list must be expanded to include UPOs that are part of a commercial panel reported in 2023.^17^

Attempts to find a novel type UPO or a UPO with specific properties usually require extensive screening work. This is even more true when mutant libraries have to be generated by random mutagenesis, which can encompass hundreds of thousands of mutants. To date, there is no screening strategy for UPOs that would be easy to implement for such large numbers of clones. The cultivation and analysis of single cell organisms such as yeasts in microtiter plates is state of the art and allows a throughput of several thousand clones at best.^17,18^

A higher throughput with less costly laboratory equipment can be achieved if UPO-secreting cells are identified directly on agar plates. A suitable substrate for the detection is 2,2′-azino-*bis*(3-ethylbenzothiazoline-6-sulfonic acid) (ABTS) that is oxidized by the peroxidase activity of UPOs (one-electron oxidation) resulting in the formation of a semi-stable cation radical with an indicative blue-green colour.^19^ Since UPOs strictly rely on hydrogen peroxide for their reaction (and the transformed hosts are not expected to form extracellular H_2_O_2_), the co-substrate needs to be provided externally. Very recently, Schmitz et al. have reported an agar plate-based UPO activity assay^20^ using *Pichia pastoris* (syn. *Komagataella phaffii*), a yeast that is frequently used as the production host for UPOs due to its high protein yields.^17,21–25^ On the other hand, the transformation efficiency for *P. pastoris* is rather low, especially when using the standard lithium method.^26^ Therefore, this yeast is not the organism of choice for mutant screenings involving large numbers of clones, and thus, we focussed here on *Saccharomyces cerevisiae*, which is a common expression host for various recombinant proteins including UPOs.^18,27^ It is particularly suitable as a biological screening tool as its transformation efficiency is relatively high^28,29^ and its propensity for homologous recombination facilitates cost-effective and relatively simple cloning methods.^30^

RETRACTED

Here, we present a plate-based screening procedure for UPOs recombinantly expressed in *S. cerevisiae* that enables the highest throughput to date. In order to realize the above-mentioned supply with the co-substrate H_2_O_2_, we modified the standard ABTS-agar for the detection of laccase and peroxidase activities. In this way, two previously undescribed short UPOs could be identified from an exemplary library of putative UPO genes. The subsequently produced and characterized UPOs show interesting catalytic properties with regard to the *in vitro* synthesis of human drug metabolites.

## Materials and methods

All chemicals were purchased from Sigma-Aldrich, Schnelldorf, Germany and were of reagent-grade purity, unless otherwise stated. Additional methods with corresponding references are described in the supplementary material section.

### Plasmids

The plasmids used in this study are based on the commercial pYES2-vector (Thermo Fisher Scientific, Germany). The genes for the putative UPOs tagged with a C-terminal 6×His-peptide were synthesized and cloned into pYES2 by GeneArt (Thermo Fisher Scientific, Germany). The yeast adapted mutant PaDa-I of *Aae*UPO,^18^ also cloned into pYES2, served as the positive control for the proof of concept.

### Selection of putative UPO genes

A small library comprising 20 genes of putative UPOs from the subfamily I.5, which includes well-characterized UPOs (e.g., *Marasmius rotula*, *Leptoxyphium fumago*, *Hypoxylon* sp.), was assembled by searching the NCBI database. The focus was on sequences from different fungal phyla (Ascomycota and Basidiomycota) as well as with different lifestyles (saprotroph, phytopathogenic, wood-associated, leaf-associated). Since many of these sequences are derived from genome sequencing projects, a stringent filtering for correctly coding sequences was applied, which included searches for incorrectly predicted introns and necessary UPO specific motifs. Subfamily I.5 contains short UPOs with a mean size of 29 kDa, the highly conserved -PCP- motif and the -EHD-S-E- motif that is specific for short UPOs.^5^ To gain extracellular enzymes, only sequences with secretion signals that were identified with SignalP5.0 were considered.^27^ The UPO genes selected are listed with their respective accession numbers in Table S1. For expression, the corresponding open reading frames (ORF) were designed with a codon usage that was optimized for *S. cerevisiae*. Sequences were aligned using Clustal Omega 1.2.2^28^ and a maximum likelihood phylogenetic analysis was performed using PhyML 3.3.20180214^29^ including 200 bootstrapping replicates to calculate branch support.

RETRACTED

### Transformation of *S. cerevisiae*

The preparation of competent cells of *S. cerevisiae* INVSc1 and the transformation of them with autonomously replicating plasmids was carried out as reported in the protocol of Gietz and Schiestl.^28^ The amount of plasmid DNA used for the transformations of the controls in the initial experiments was between 200 and 300 ng. For the screening, the plasmids containing the putative UPO genes were pooled. In the transformation mix, each plasmid had a concentration of 5 ng µL^−1^. After transformation, cells were plated on agar containing SC minimal medium without uracil (5 g L^−1^ ammonium sulphate, 1.7 g L^−1^ YNB w/o amino acids and w/o ammonium sulphate, 1.92 g L^−1^ yeast synthetic dropout w/o uracil, 15 g L^−1^ agar) and with 20 g L^−1^ glucose, and grown at 30 °C for 3 days.

### ABTS-based plate screening

The general procedure for the ABTS-based plate screening is described here for the above-mentioned screening of the plasmid pool. The yeast colonies grown on SC minimal medium agar without uracil and with glucose after the transformation were collected as a cell suspension by scraping them off the plate with an inoculation loop and suspending them in 3 mL sterile desalted water. The optical density of the cell suspension was photometrically measured at 600 nm. A dilution with a concentration of 6000 cells per mL was prepared by using the equation: 1 OD_600_ correlates to 10^7^ cells mL^−1^.^28^ 400 µL of the corresponding cell suspension was plated on a 14 cm Petri dish containing 50 mL SC minimal medium agar (0.5 cm bottom layer) with 20 g L^−1^ of the inducer substrate galactose instead of glucose and 0.6 mM of the indicator ABTS. As top layer, 30 mL of the same medium, but with only 0.7 g L^−1^ agar and still liquid (at a temperature of 40 °C), was poured onto the bottom layer so that the yeast cells were embedded. The plates were incubated at 30 °C for 5 days. For the detection of ABTS radicals formed by secreted UPOs, 3 mL 20 mM hydrogen peroxide were spread on the top layer and incubated for at least 20 min at room temperature. Colonies with blue-green zones were picked with a toothpick and transferred to fresh agar plates containing SC minimal medium with 20 g L^−1^ glucose.

RETRACTED

### Colony PCR and sequencing

To identify the UPO genes responsible for the ABTS-positive reaction in the plate tests, the corresponding region on the plasmid was amplified from the potential hits by colony PCR. From each colony, a small amount was suspended in 50 µL of 1×TE buffer with 50 U mL^−1^ Yeast Lytic Enzyme from *Arthrobacter luteus* (Thermo Fisher Scientific, Germany), incubated at 37  °C for 30 min and heat inactivated at 95  °C for 10 min. The PCR was performed with the Hot Start Taq 2× Master Mix (NewEngland Biolabs) and 1 µL of the lysate according to the manufacturer's manual. The PCR products were purified with the Monarch PCR & DNA Cleanup Kit (NewEngland Biolabs) according to the manual. Sanger sequencing of the amplicons was done by LGC Genomics GmbH (Berlin, Germany).

### Production and characterisation of recombinant UPOs (rAniUPO and rDbiUPO)

*S. cerevisiae* INVSc1 was freshly transformed with the plasmids containing the UPO genes of *Aspergillus niger* (*Ani*UPO) and *Dendrothele bispora* (*Dbi*UPO), after their identification as the positive hits. For enzyme production, a colony of both yeast clones was used for inoculating 500 mL baffled flasks containing 100 mL SC minimal medium with 20 g L^−1^ glucose. The flasks were incubated at 30 °C and 200 rpm for three days. 50 mL of these precultures were transferred to fresh 1 L baffled flasks, containing 150 mL expression medium (30 g L^−1^ galactose, 5 g L^−1^ ammonium sulphate, 1.7 g L^−1^ YNB w/o amino acids and w/o ammonium sulphate, 1.92 g L^−1^ yeast synthetic dropout w/o uracil, 140 mM potassium phosphate buffer pH 6.0, 1.17 g L^−1^ MgSO_4_, 0.42 g L^−1^ FeSO_4_, 3.3% ethanol, 25 mg L^−1^ chloramphenicol). The cultures were incubated at 24 °C and 200 rpm for six days. Supernatants were separated from the cells by centrifugation at 5000 g for 20 min and concentrated using a SartoJet ultrafiltration device (Sartorius AG, Göttingen, Germany) with a 10-kDa cut-off membrane. Further concentration was accomplished with a Minimate^TM^ TFF system (Pall Corporation, New York, USA) with the same cut-off.

### Enzyme assays

In order to use adequate amounts of active r*Ani*UPO and r*Dbi*UPO in the enzymatic tests, the enzyme concentration in the concentrated culture supernatants was calculated using corresponding carbon monoxide difference spectra.^31^ Briefly, a cuvette was filled with 1440 µL 50 mM potassium phosphate buffer (pH 7.3), 400 µL 300 mM Na_2_S_2_O_4_ (dissolved in 1.3 M potassium phosphate buffer, pH 8.0) and 160 µL enzyme solution. The spectrum was recorded between 400 and 500 nm with a photometer (BioMate™ 160 UV/VIS photometer, Thermo Fisher Scientific, Germany). Then, the cuvette was flushed with carbon monoxide (CO) at a constant flow rate (one bubble per second). Afterwards, the spectrum was recorded again. The CO absorption maximum of the UPOs was at 444 nm. The concentration of active UPO was calculated as described by Otey.^31^

RETRACTED

The catalytic profile of r*Ani*UPO and r*Dbi*UPO was characterized by the conversion of following substrates: propranolol, diclofenac, testosterone, eicosapentaenoic acid (EPA), docosahexaenoic acid (DHA) and clopidogrel. Reactions (100 μL total volume) were initiated by adding 90 μL of the reaction mixture (1 mM substrate, 1 mM hydrogen peroxide, 5 mM ascorbate, 20 mM potassium phosphate buffer, pH 7.0) to 10 μL of a 4.5 µM UPO solution. The reaction mixtures were incubated at 25 °C and 800 rpm on a thermal shaker (TurboShaker 3500, Scienova GmbH, Jena, Germany) for 30 min and stopped by the addition of 100 μL of ice-cold acetonitrile (−20  °C). Subsequently, the samples were centrifuged at 14,000 g for 10 min, the supernatants were transferred into HPLC vials and analyzed by liquid chromatography-mass spectrometry (LC-MS/MS) as described previously.^32^

In addition to the above substances, the oxidation of the prototypical UPO substrates veratryl alcohol (VA), 2,2′-azino-*bis*(3-ethylbenzothiazoline-6-sulfonic acid) diammonium salt (ABTS), 5-nitrobenzodioxole (NBD) and 2,6-dimethoxyphenol (DMP) was assayed photometrically according to^19^ in appropriate cuvette tests. The added UPO concentration was 4.5 µM and the formation of veratraldehyde (ε_310_= 9300 M^−1^ cm^−1^), the ABTS cation radical (ε_420_= 36,000 M^−1^ cm^−1^), 5-nitrocatechol (ε_425_= 9700 M^−1^ cm^−1^) and coerulignone (ε_469_= 27,500 M^−1^ cm^−1^) was monitored using a BioMate™ 160 UV/VIS photometer (Thermo Fisher Scientific, Germany).

## Results

### Phylogeny of a selection of putative UPO genes

The UPO sequences selected for the screening library were from the fungal phyla Ascomycota and Basidiomycota, and belonged only to the subfamily I.5 (short UPOs)^9^ (Figure 1).

**Figure 1.** Maximum likelihood tree of the putative short UPO sequences selected for the screening library. Phylogeny was calculated using PhyML 3.3.20180214 with a log-likelihood score of −10174.09410. Branch support was estimated using 200 bootstrap replicates; only support >90% were shown above branches. The outgroup UPO sequence is from *Rozella allomycis* (Cryptomycota), the evolutionary oldest group of fungi (Eumycota).

RETRACTED

The phylogenetic tree reveals two clusters, one of which contains both ascomycetous and basidiomycetous sequences (the latter forming a separate sub-cluster), while the other contains only ascomycetous sequences. Furthermore, it is evident that the sequence of the long-known chloroperoxidase from *Leptoxyphium (Caldariomyces) fumago*, which formally belongs to the short peroxygenases, shows particularly strong deviations (evolutionary distance) from the other UPOs.

#### ABTS-based plate screening

To evaluate the plate-based activity screening with *S. cerevisiae*, the method was tested using an established strain of this species as a positive control, which expresses the mutant clone PaDa-I of the model UPO from *Cyclocybe (Agrocybe) aegerita* (*Aae*UPO) with high efficiency;^18^ a strain with an empty vector served as a negative control. Mixtures of cell suspensions were prepared containing about 2% or 10% cells bearing the UPO gene amidst a majority of UPO-negative cells. Over the time course of several days, the cells, plated on agar containing the inducer galactose and the indicator substrate ABTS, grew well embedded in the “soft agar” (Figure 2). To visualize extracellular UPO activity, the co-substrate H_2_O_2_ was spread as a thin aqueous film on the top layer. Over a period of about 15 min, the hydrogen peroxide diffused into the agar and the characteristic blue-green color of the ABTS cation radical developed around some of the colonies. In the tests shown in Figure 2, the actual number of positive colonies was approximately equal to the calculated number, i.e., 5 out of 96 colonies for the plate with 2% of UPO-containing cells and 8 out of 74 for the 10% mixture. The majority of the colonies, however, did not show any color change and remained white.

**Figure 2.** Evaluation of an ABTS-based plate screening for UPO-secreting *S. cerevisiae* colonies. *S. cerevisiae* cells containing a plasmid with the positive control *Aae*UPO PaDa-I were mixed with cells that contained the empty vector at a ratio of 1:50 (2%, left) or 1:10 (10%, right). UPO-positive colonies developed blue-green zones caused by the oxidation of ABTS after addition of H_2_O_2_.

Once the method had been validated, its applicability was proven by testing the above library containing a selection of short UPO genes. *S. cerevisiae* was transformed with a pool of 20 plasmids and a fraction of this transformation mix was spread onto agar plates with glucose. 455 colony-forming units (cfu) were obtained after 3 days, representing a 22-fold coverage of the plasmid pool. These colonies were scraped from the agar plates, suspended in water and a fraction was re-plated on agar with the expression medium and subsequently covered with a layer of “soft agar”. Approximately 4000 cfu grew on the screening plates, and after 5 days growth and addition of hydrogen peroxide, approx. 40 colonies developed dark blue-green colored zones. Almost the same number of colonies produced a less intensive color reaction (Figure 3). However, the size of the colored zones was significantly smaller than in the established positive control *Aae*UPO PaDa-I (Figure 2).

RETRACTED

**Figure 3.** Screening for activity of extracellular UPOs recombinantly expressed in *S. cerevisiae*. A pool of 20 putative UPO ORFs was screened using a plate-based approach with ABTS as indicator. Color formation caused by the UPO catalyzed oxidation of ABTS developed after addition of H_2_O_2_. The picture on the right shows a close-up of the plate.

Of these colored colonies, 19 were selected to identify the responsible UPO genes. Sanger sequencing revealed that 14 of them corresponded to a UPO from *Dendrothele bispora* (*Dbi*UPO; accession number THU92580) and two to a UPO from *Aspergillus niger* (*Ani*UPO; accession number XP_001390900.2). The quality of the remaining three sequencing results was insufficient for further evaluation.

#### UPO production and substrate portfolio

*S. cerevisiae* cells were freshly transformed with plasmids containing the genes of *Ani*UPO or *Dbi*UPO. In order to optimize enzyme production, media with varying compositions were tested as exemplarily shown for r*Ani*UPO (Figure 4). The best result in terms of active recombinant protein was achieved by a combination of increased amounts of galactose, Fe^2+^ and Mg^2+^ ions. The volume activity in the untreated supernatants of cultures containing r*Ani*UPO was highest on the fifth day of cultivation and amounted to 730 U L^−1^, measured with ABTS as substrate (Figure 5). In the case of r*Dbi*UPO, the volume activity was significantly lower (≤ 5 U L^−1^).

**Figure 4.** Influence of different medium compositions on the production of r*Ani*UPO in the host *S. cerevisiae* INVSc1. The volume activity in the supernatants was monitored over the cultivation period with ABTS as substrate; media composition and the abbreviations in the legends are given in table S2.

**Figure 5.** Monitoring the enzymatic volume activity in the supernatants of *S. cerevisiae* INVSc1 producing r*Ani*UPO or r*Dbi*UPO. Enzyme activity was measured with ABTS as substrate. Cultivations were carried out in duplicate.

The concentrated supernatants containing the recombinant UPOs were used to analyze the conversion of prototypical UPO substrates photometrically (Table 1) and of selected pharmaceuticals and PUFAs (Table 2) by LC-MS/MS. An analogously treated supernatant from a culture, which did not express UPO activity, served as control and showed no activity towards the tested substrates.

RETRACTED

**Table 1.** Oxidation of prototypical UPO substrates by r*Dbi*UPO and r*Ani*UPO. Product formation was determined photometrically. Enzyme activities are given in U mL^−1^. Equal concentrations of active UPO protein were applied based on the calculation from the corresponding CO-difference spectra. Data are means ± SD with n = 3.

Substrate	Mode of action/type of reaction	r*Ani*UPO	r*Dbi*UPO
ABTS	one-electron oxidation of a non-phenolic substrate^15^	5.9 ± 0.09	11.9 ± 0.55
VA	peroxygenase activity, i.e., alcohol oxidation via hydroxylation and release of water^29^	0.7 ± 0.04	4.1 ± 0.27
DMP	one-electron oxidation of a phenolic substrate^15^	3.5 ± 0.01	3.0 ± 0.04
NBD	*O*-dealkylation (demethylenation) via hydroxylation and formate release^15^	0.8 ± 0.08	0.4 ± 0.04

**Table 2.** Conversion of pharmaceuticals and polyunsaturated fatty acids (PUFAs) by r*Dbi*UPO and r*Ani*UPO. 0.45 M enzyme was used to convert 1 mM substrate in the presence of 5 mM ascorbate and 20 mM potassium phosphate buffer, pH 7.0. The reactions were started by the addition of 1 mM H_2_O_2_ and incubated at 25°C for 30 min. Oxidation of propranolol (**1**), diclofenac (**2**), testosterone (**3**), eicosapentaenoic acid (EPA; **4**), docosahexaenoic acid (DHA; **5**) and clopidogrel (**6**) was analyzed by LC-MS/MS and a selection of relevant products is given. Turnover frequency (TOF) per hour (h^−1^) is displayed for all substrates in the second column below the enzyme abbreviations. The formed products (numbers in brackets) are listed in table S3, stacked LC-MS/MS chromatograms from TIC and EIC as well as MS/MS spectra are depicted in figure S3–S8 in the supplementary material.

Both enzymes were able to oxidize the four typical UPO substrates, though to different extent in dependence of the particular substrate. r*Dbi*UPO showed the highest activity towards ABTS followed by veratryl alcohol (VA), 2,6-dimethoxyphenol (DMP) and 5-nitrobenzodioxole (NBD), while r*Ani*UPO followed the order ABTS > DMP > NBD ∼ VA.

Mass analyses of products focused on those that are relevant as human (drug) metabolites.^12–14,33,34^ For all tested substrates, the formation of oxygenated products could be observed by an indicative mass increase of 16 m/z compared to the original masses (for details, see Supplementary Material). In the case of EPA and DHA, the incorporation of more than one oxygen atom was observed in addition to single oxygenation.

RETRACTED

## Discussion

When searching for new or modified biocatalysts, it is essential to find the right screening strategy. Agar-plate based methods are widely used for the identification of various enzymes, not least because they are inexpensive and simple.^35^ In this study, such a method was established for the screening of secreted fungal UPOs recombinantly expressed in the host yeast *S. cerevisiae*. UPOs require hydrogen peroxide as co-substrate (electron acceptor and oxygen source) for action, which cannot be supplied by the yeast and therefore has to be provided externally. It is inevitable that colonies grown on an agar plate will mix when the liquid cosubstrate is applied. To prevent this, we grew the cells/colonies here embedded in an additional agar layer which kept the colonies separated even after the addition of hydrogen peroxide. *S. cerevisiae* showed no interfering background activities (e.g., by intrinsic peroxidases or multicopper oxidases) towards the indicator substrate ABTS. Thus, hits (UPO-positive colonies) could be easily detected and picked, and the method as such proved to be reliable and easy to handle. Schmitz et al.,^20^ who developed a similar detection method for the UPO host *P. pastoris*, reported that it can even be performed semi-quantitatively. We can confirm this finding, since *S. cerevisiae* colonies that secrete the well-adapted recombinant PaDa-I variant of *Aae*UPO^18^ produced larger and more intensively colored zones than the non-optimized positive UPOs in our library screening. To prove the applicability of the agar plate-based method, a library of 20 gene sequences of short UPOs with different phylogenetic background was studied. Due to the good transformation efficiency of *S. cerevisiae*, a more than 20-fold coverage of the plasmid pool could be achieved.

Two hits were identified from the library. One sequence belongs to a UPO from *Dendrothele bispora*, an unusual member of the basidiomycetous class Agaricomycetes (family Marasmiaceae), whose fruiting body is not piliate-stipitate (i.e., with stalk and cap) but crust-like as those of many wood-rot fungi.^36^ Its correct taxonomic position within the family Marasmiaceae was confirmed here by the high sequence homology (54%) of its UPO with that of the model fungus *Marasmius rotula* (compare Figure 1).^37^ The other sequence is from *Aspergillus niger*, a well-known and widely used ascomycetous mold of the class Eurotiomycetes.^38^ It was derived from a set of six UPO sequences already studied by Rotilio et al. 2021,^24^ who also examined the corresponding UPO proteins with regard to their activities, but using a special strain of *P. pastoris* for expression. They detected UPO activities for all six candidates in *P. pastoris* cultures but reported on stability problems (heme loss) when the enzyme production was up-scaled (only one UPO from a *Hypoxylon* sp. strain could be obtained in sufficient amounts). In contrast, the only enzyme from this sequence set that was actively expressed in our approach with *S. cerevisiae* was *Ani*UPO (accession number XP_001390900.2). The explanation for the different outcomes could lie in the use of a different host yeast. There are reports on the expression of UPOs in yeasts where *P. pastoris* was a better host than *S. cerevisiae* in terms of protein yields, albeit not in all cases.^39^ Moreover, we were working with a different genetic background here. The studied UPOs were expressed with their native signal peptides, whereas Rotilio et al. fused the mature UPO to an artificial signal peptide. This might have an impact on the translational level as well as on the secretion process.^23,39^ Finally, all UPOs tested here were provided with a C-terminal polyhistidine fusion tag to facilitate purification. In the case of *Aae*UPO PaDa-I, such modification was shown to affect activity,^40^ and may have masked the UPO secretion that occurred in our plate-based screening.

RETRACTED

Both r*Ani*UPO and r*Dbi*UPO were capable of converting pharmaceuticals and PUFAs into metabolites that are relevant in the human body, albeit with different regioselectivities and efficiencies. Propranolol (**1,** see Table 2), a widely used drug and typical UPO substrate for drug oxyfunctionalization,^41^ was oxidized to 4-hydroxypropranolol (**8,** see Table 2) and 5-hydroxypropranolol (**7,** see Table 2). The hydroxylation pattern differed between the two enzymes, where r*Ani*UPO produced mostly (**8,** see Table 2), while r*Dbi*UPO formed both aromatic isomers. In the case of diclofenac (**2,** see Table 2), it was shown that both UPOs tend to form 4-hydoxydiclofenac (**9,** see Table 2), while the formation of the isomeric form 5-hydroxydiclofenac (**10,** see Table 2) was limited. This indicates that the enzymes preferably activate halogenated aromatic rings through oxygenation.^42^ The reaction with testosterone (**3,** see Table 2) led to a monooxygenation at an uncertain position (**11,** see Table 2) but only in the case of r*Ani*UPO, while r*Dbi*UPO failed to oxygenate this bulky molecule. Similar observations have been made for various other enzymes including UPOs with narrow or less affine substrate channels.^33,43–46^ Therefore, it can be concluded that r*Dbi*UPO has a rather small and hydrophobic substrate pocket and/or heme access channel. This assumption was supported by the results on PUFA conversion, in which EPA (**4,** see Table 2) and DHA (**5,** see Table 2) were first monooxygenated by both enzymes, but later only further oxygenated by r*Ani*UPO. In both cases, a single incorporation of an oxygen atom (**12**, **15,** see Table 2) was accomplished, while a double and even triple oxygen insertion (**13**, **14**, **16**, **17,** see Table 2) was preferably and exclusively realized by r*Ani*UPO. This indicates that the monooxygenated product no longer fits into the substrate channel/pocket of r*Dbi*UPO after the increase in polarity and size due to oxygen incorporation, resulting in a constricted active site.^47^

RETRACTED

Clopidogrel was used as a potential multi-target substrate, for which the ability of the rUPOs was tested to catalyze sequential oxygenations/oxidations.^14^ The formation of the oxidation product 2-oxo-clopidogrel (**18,** see Table 2) was demonstrated for both enzymes, just as the dimerization of two sulfoxide derivatives resulting from the initial *S*-oxygenation of two clopidogrel molecules (**19,** see Table 2). The most interesting metabolite of clopidogrel is the ring-opening product (**20,** see Table 2), which has been described as an effective antiplatelet drug (antiaggregant).^48^ This molecule may originate from the cleavage of (**18,** see Table 2) that is a thiolactone. As this was only observed for r*Ani*UPO, it indicates an oxygenolytic activity on **18**, which is diminished or missing in r*Dbi*UPO. In general, product yields for r*Dbi*UPO were lower in most cases, although this might not essentially be attributed to lower substrate conversion, but also to the formation of unknown products. A reason for this could be that some of the products formed by r*Dbi*UPO did not result from the peroxygenase activity that would insert peroxide-borne oxygen into the substrates, but also from the peroxidase activity, which may produce radicals that tend to spontaneous coupling reactions.^8^ This assumption is consistent with the results of tests with typical UPO substrates, where the enzyme tended to have peroxidase rather than peroxygenase activities. It is also in accordance with recent results on another short UPO from *Dendrothele bispora* (accession number: THV03356.1),^17^ which shows 65% sequence homology to our r*Dbi*UPO. From the substrate spectrum of this enzyme, it was deduced that r*Dbi*UPO has a narrow substrate channel, which hinders the direct access of larger substrate molecules to the heme and thus preventing peroxygenase activity (oxygen transfer). On the other hand, our ligand-protein-docking studies with the enzyme and diclofenac as representative substrate did not confirm this assumption (Figure S7 in the Supplementary Material). It can therefore not be ruled out that the results are due to the above-mentioned interference by the C-terminal His-tag. Such a tag could be more severe for r*Dbi*UPO than for r*Ani*UPO. There are UPOs that exist as functional homodimers such as the main UPO from *Marasmius rotula,*^49^ in which the dimer is formed by bridged cysteine residues at the C-termini. A similar cysteine is present in the related *Dbi*UPO (compare Figure 1), but not in *Ani*UPO, and the polyhistidine-tag could have a detrimental effect on the disulfide bond and hence on functional dimer formation.

RETRACTED

In summary, two new functional UPOs were identified using the plate-based screening method. r*Dbi*UPO is particularly suitable for the synthesis of monooxygenated products, e.g., from polyunsaturated fatty acids, while r*Ani*UPO is the better candidate for the preparation of (poly)hydroxylated and carbonylated metabolites from bulkier substrates.

## Conclusion

The search for new recombinant UPOs is a useful attempt as shown in the present study. The enzymes found have different catalytic properties with regard to their substrate preferences and product patterns, and may be therefore suitable for different types of application. The established plate-based screening approach for recombinant UPOs produced in *S. cerevisiae* has proven to be a fast, simple, yet reliable high-throughput method that requires little technological effort. Although the assay was initially developed using ABTS as an indicator, it can be expanded to other chromogenic or fluorescent substrates (or their products) to look for a particular specific activity. The high number of clones that can be examined at once makes it suitable for the screening of large libraries, for example, from random mutagenesis approaches. The scope of this method should not be limited to the search for new expressible UPOs, but could also be used for the identification of UPOs with specific properties, such as thermostable mutants.

## Supplemental Material

sj-docx-1-chm-10.1177_13860291241306566 - Supplemental material for Rapid screening system to identify unspecific peroxygenase activity Supplemental material, sj-docx-1-chm-10.1177_13860291241306566 for Rapid screening system to identify unspecific peroxygenase activity by Marina Schramm, Carlos Renato Carrillo Avilés, Johannes Kalmbach, Kai-Uwe Schmidtke, Jan Kiebist, Harald Kellner, Martin Hofrichter and Katrin Scheibner in Clinical Hemorheology and Microcirculation
